# Association between brain morphometry and aerobic fitness level and sex in healthy emerging adults

**DOI:** 10.1371/journal.pone.0242738

**Published:** 2020-12-01

**Authors:** Natasha E. Wade, Alexander L. Wallace, Ryan M. Sullivan, Ann M. Swartz, Krista M. Lisdahl

**Affiliations:** 1 Department of Psychiatry, University of California, San Diego, CA, United States of America; 2 Department of Psychology, University of Wisconsin-Milwaukee, Milwaukee, WI, United States of America; 3 Department of Kinesiology, University of Wisconsin-Milwaukee, Milwaukee, WI, United States of America; Nuovo Ospedale Prato (NOP) Santo Stefano, USL Toscana Centro, ITALY

## Abstract

**Objective:**

Aerobic fitness may be beneficial for neuroanatomical structure. However, few have investigated this in emerging adults while also accounting for potential sex differences. Here we examine aerobic fitness level, sex, and their interaction in relation to cortical thickness, surface area, and volume.

**Method:**

Sixty-three young adults between the ages of 16–26 were balanced for sex and demonstrated a wide range of aerobic fitness levels. Exclusion criteria included left-handedness, past-year independent Axis-I disorders, major medical/neurologic disorders, prenatal medical issues, prenatal alcohol/illicit drug exposure, or excessive substance use. Participants completed an MRI scan and a graded exercise test to volitional fatigue (VO_2_ max). Data analyses were run in Freesurfer and data was corrected for multiple comparisons with Monte Carlo simulations at .05.

**Results:**

Males demonstrated higher VO_2_ values. Higher VO_2_ values were statistically independently related to thinner lateral occipital, superior parietal, cuneus, precuneus, and inferior parietal regions, smaller lateral occipital volume, and larger inferior parietal surface area. Compared to females, males had larger volume in rostral anterior cingulate, lateral occipital, and superior frontal regions, and greater surface area in fusiform, inferior parietal, rostral and caudal anterior cingulate, and superior parietal regions. VO_2_*Sex interactions revealed higher-fit females had higher inferior parietal, paracentral, and supramarginal surface area, while lower-fit males showed larger surface area in these same regions.

**Conclusions:**

Individuals with higher aerobic fitness performance had thinner cortices, lower volume, and larger surface area in sensorimotor regions than lower fit individuals, perhaps suggesting earlier neuromaturation in higher fit individuals. Larger surface area was associated with higher-fit females and lower-fit males. Thus both sex and aerobic fitness are important in shaping brain health in emerging adults.

## Introduction

Adolescence and young adulthood is marked by extensive neurodevelopment. Gray matter changes tend to follow a U-shaped curve [1], as gray matter volume first grows throughout childhood and then, subsequently into adolescence and emerging adulthood, reduces as pruning eliminates unnecessary or inefficient connection. The natural trajectory of these maturational processes are likely impacted by external factors, such as through physical exercise (see [2], for review). However, studies thus far have only limitedly considered the impact of aerobic fitness level on cerebral structure. Further, as sex influences aspects of neurodevelopment [3], it is important to consider sex differences in the association between aerobic fitness and gray matter morphometry.

Brain health and structure can be measured through a number of methods. In particular, gray matter is often used to measure subtle changes in neural maturation in the developing brain. Gray matter volume, surface area, and thickness are means of assessing developmental trajectories across the lifespan [1,4,5]. Following a burst of growth, measures of gray matter volume often reduce, indicating maturation through pruning [6]. Along the same timeframe, cortical thinning occurs through a linear trajectory, while surface area follows a cubic curve throughout adolescence [7]. While most measures demonstrate unique trajectories by sex [8,9], cortical thickness appears to be less influenced by sex [10].

Aerobic fitness, including increases in fitness through aerobic exercise routines, has been linked to a number of factors that likely influence neurodevelopment. Moderate intensity aerobic exercise has been shown to result in greater neurogenesis in animals compared to high-intensity interval training [11] or resistance training [12], as well as proposed in humans [13], suggesting increased fitness may similarly relate to more neurogenesis. Brain-derived neurotrophic factor (BDNF), vascular growth factors, and other growth factors increase in response to exercise and improved fitness level [14–19]. Catecholaminergic function, too, appears to be positively impacted by exercise [20,21]. Neural inflammation may also be reduced following exercise and increased activity of growth factors [14,22], further suggesting another mechanism by which aerobic exercise and, in turn, fitness may benefit brain development.

Such multi-factorial mechanisms may explain the proposed beneficial influence of aerobic fitness level on brain health. In multiple studies of healthy adolescents and young adults, changes in BDNF and reduced inflammatory response was related to better performance on cognitive tasks in individuals with higher aerobic capacity [23,24]. Larger volumes in subcortical and frontal regions have been related to higher aerobic fitness in children and adolescents [25–29]. Similarly, thinner cortices were found in higher fit children, adolescents, and young adults across the cortex [30,31]. Larger surface area of the right medial pericalcarine, right cuneus, and left precuneus related to fitness in male teens [27], thinner cortices in posterior cingulate and supramarginal cortices in young adults [31], and larger volumes in regions such as the PFC and parietal lobe, amongst others [29]. Morphometrical associations between regions such as the PFC and parietal cortex and fitness may then represent age-appropriate optimal pruning [32,33]. These macrostructural changes also likely impact function, as has been shown in several studies [25,26,29,30,34], and are predictive of performance over time [35]. These prior works suggest a positive relationship between aerobic fitness level and brain morphometry.

Importantly, the vast majority of the literature on neurodevelopment in relation to aerobic fitness so far has focused on prepubescent youths or, when including adolescents, males. As brain development continues well into an individual’s 20’s, it is also important to investigate these relationships into young and emerging adulthood. Further, no known studies have specifically assessed sex in relation to neuroanatomy and fitness in adolescents and young adults. Most studies have only included males [27,28,36] or controlled for sex [29,31], which does not allow for addressing potential sex-related differences in neuroanatomical structure, despite differences in VO_2_ performance by sex [29]. This is important as sex may also play an important moderating role between aerobic fitness or exercise and brain-behavior outcomes. Highly fit females demonstrate better executive function compared to low-fit females [37] and female IQ scores increase with aerobic exercise intensity compared to men [38]. Sex influences the effect of aerobic exercise on BDNF levels, and respiratory and cardiovascular systems [39]. Females also peak in neuroanatomical volumes approximately 1–2 years before males [9]. Given neuroanatomical characteristic differences by age *and* sex [8,9] and potential differences in underlying neuromechanisms, it is important to consider the influence of these factors in any neuroimaging developmental study.

Thus, the present study aims to assess the relationship between aerobic fitness, measured objectively by graded exercise testing, and neuroanatomical structural characteristics in healthy adolescents and young adults without evidence of metabolic disorders. Based on prior findings, we generally expected to see larger volumes [27,29], thinner cortices [31], and larger surface area [27] associated with higher fitness level in prefrontal and parietal regions in late adolescents and young adults [32,33]. In addition, we conducted exploratory analyses to assess whether sex interacted with aerobic fitness level in relation to neuroanatomical morphometry.

## Materials and methods

### Participants

Local newspaper advertisements and fliers in Milwaukee, Wisconsin were used to recruit sixty-three healthy emerging adults (36 low-fit, 27 high-fit). Fitness groups were created based on VO_2_ performance during study sessions, with individuals performing at or above the 50^th^ percentile for their age and sex [40] being considered high-fit, and all others being considered low-fit. Groups were used to understand participant demographics, but continuous variables of VO_2_ values were used in all analyses.

Participants were between the ages of 16 and 25y (M = 21.2, SD = 2.6), were sex balanced (50.8% female), and predominately Caucasian (69.8%). Participants were included if they were right handed, spoke English, and were willing to abstain from any substance use over a 3-week period. Exclusion criteria included having an independent DSM-IV Axis I (attention, mood, anxiety, or psychotic) disorder in the past year, major medical (including hyperlipidemia, hypertension or diabetes) or neurological disorders, no loss of consciousness >2 minutes, prenatal medical issues or premature birth (gestation <35 weeks), reported prenatal alcohol/illicit drug exposure, or excessive other drug use (>20 times of lifetime use for each drug category).

### Procedures

Data was used from a larger parent study examining the neurocognitive effects of cannabis use in youth (R01 DA030354; PI: Lisdahl); all aspects of the protocol were IRB-approved and in accordance with the Declaration of Helsinki. Potential participants who expressed interest in the parent study were screened through an initial brief phone screen to confirm basic study criteria and then provided written consent/assent through the mail for a semi-structured interview over the phone (see Detailed Phone Screen below). If determined eligible, study staff obtained written consent from participants (aged 18 or older). All minors below 18 years of age provided written assent after parent consent was obtained. Parents of participants were consented for a parent-administered phone interview that screened for medical, psychiatric and prenatal history. Participants who were eligible for the study came in for five study sessions over the course of three weeks. The first three sessions occurred one week apart and consisted of urinary drug analysis and a brief neuropsychological battery (data presented elsewhere; see [41]). Session 4 occurred one week later and included self-report measures, a 3-hour neuropsychological battery (data presented elsewhere; see [42] for full battery) and VO_2_ performance testing. Session 5 was conducted within 24–48 hours of Session 4 and consisted of MRI scanning. Across study sessions, participants were asked to remain abstinent from alcohol, cannabis, and other drug use, which was confirmed through breath, urine and sweat toxicology screening. If positive for any drug or having a breath alcohol concentration greater than .000 at the start of Session 4 (neuropsychology battery and VO_2_ testing) or Session 5 (MRI scan), participants were deemed ineligible for study participation. While nearly all participants in the parent study completed each aspect of the protocol, only healthy individuals who met the above listed inclusion/exclusion criteria were included in the present analyses.

The University of Wisconsin-Milwaukee and Medical College of Wisconsin institutional review boards approved of all aspects of this study (IRB Protocol Number: PRO0001602).

### Measures

#### Detailed phone screen

Following initial screening, written assent/consent was obtained from each participant and parent via mail. A 45-minute detailed phone screen was then scheduled and conducted. ***Mini Psychiatric Interview***—Participants and parents of minors were interviewed using the Mini International Psychiatric Interview (MINI) [43] or MINI-Kid [44] to screen out for psychiatric comorbidities. ***Lifetime substance use***—To determine lifetime patterns of drug and alcohol use, youth participants were given the Customary Drinking and Drug Use Record (CDDR) [45] at baseline to measure frequency of alcohol, nicotine, cannabis, and other drug use (i.e., cocaine, methamphetamine, MDMA/ecstasy, heroin, taking medications without a prescription, GHB, psilocybin, hallucinogens, salvia, inhalants, steroids, or any other reported substance use), SUD symptoms, and the age of onset for first time and regular (weekly) use.

#### Substance use

Past-year substance use was measured using the Timeline Follow-Back (TLFB; [46,47]). Standardized units of cannabis (joints), alcohol (standard drinks), and other drug use for the past year was calculated using a calendar and cueing participants to significant events (memories, holidays, birthdays, etc.).

As noted in the exclusion criteria, participants were excluded for excessive other drug use (>20 episodes in their lifetime for each drug category). In addition, included participants reported substance use that is consistent with age-based normative use (e.g., in the past year, 200–240 standard drinks [48]) or lower than in studies of emerging adult substance use (e.g., 3,000 cigarettes in the past year [49] or using cannabis at least 5 days per week [50]).

#### Verifying abstinence

As participants were expected to remain abstinent from all alcohol and drugs (other han tobacco) throughout the course of the study, abstinence was evaluated at each session through urine toxicology with ACCUTEST SplitCup 10 Panel drug test and NicAlert to test cotinine level, a metabolite of nicotine, and with breathalyzer to test for alcohol use.

#### Body fat percentage

Tanita SC-331S Body Composition Monitor (Tanita, Arlington Heights, IL) was used to measure fitness characteristics, such as weight, BMI, and fat percentage. The Tanita Body Composition Monitor sent a weak electrical current from foot to foot to measure impedance throughout the body. Through this method, the amount of body fat as proportional to the participant’s body weight was measured. Additionally, body height and weight were measured using standard procedures [40].

#### VO_2_ testing

Participants were asked to refrain from food and caffeine for 4 hours prior to the exercise test. Prior to each exercise test, the metabolic measurement system, ParvoMedics TrueOne 2400 (ParvoMedics, Salt Lake City, UT) was calibrated according to the manufacturer’s instructions using a 3 Liter syringe for the pneumotachometer, and a two-point calibration for the gas analyzers (room air and a certified gas 4.08% CO_2_, 115.98% O_2_, balance N_2_). Participants were fitted with the rubber mouthpiece connected to a Hans Rudolf 2700 series two-way nonrebreathing valve (Kansas City, MO), noseclip, and heart rate strap (Polar Wearlink 31, Finland) for the collection of expired gases and measurement of heart rate. Participants completed a maximal incremental exercise test on a treadmill (Full Vision Inc., TMX425C Trackmaster, Newton, KS) following the Bruce Protocol until volitional fatigue. Expired gases were measured continuously using a ParvoMedics TrueOne 2400 metabolic measurement system (ParvoMedics, Salt Lake City, UT). Criteria for determination of attainment of VO_2_ max were based on those recommended by [51]. Metabolic data were averaged over 1 minute and exported into a spreadsheet for analysis.

### MRI methods

#### MRI acquisition

Structural MRI scans were acquired on a 3T Signa LX MRI scanner (GE Healthcare, Waukesha, WI) using a 32-channel quadrature transmit/receive head coil. High-resolution anatomical images were acquired using a T1-weighted spoiled gradient-recalled at steady-state (SPGR) pulse sequence (TR = 8.2 ms, TE = 3.4 s, TI = 450 and flip angle of 12°). The in-plane resolution of the anatomical images was 256x256 with a square field of view (FOV) of 256 mm. One hundred fifty slices were acquired at 1 mm thickness. This results in a voxel size acquisition of 1mm x 1mm x 1mm.

#### MRI data processing

Structural scans were processed through the recommended Freesurfer surface-based and volume-based reconstruction protocols [52,53]. Processing protocols consists of skull stripping and masking of the brain, registration of brain scans into MNI305 space, volumetric labeling of subcortical structures, intensity normalization to correct for intensity fluctuations across voxels, surface atlas registration, and surface extraction. All scans were visually checked by a team of three trained reviewers and manual corrections were made as needed and rerun through the reconstruction process. Quality control checks included skull stripping, segmentation, intensity normalization, pial surface placements, and any topological defects. The initial 10 scans were quality checked by all three reviewers to establish a baseline with the remaining scans, which were split between the reviewers and then checked individually. Any noted errors were brought to the reviewing team and manual edits were made accordingly by the most senior member of the team. Data was cached prior to analyses so that the chosen sample was resampled into the average subject space and smoothed at FWHM of 10.

### Statistical analyses

A series of multivariate regressions were run in FreeSurfer [54] with sex, VO_2_ levels (as a continuous measure), and sex-by-VO_2_; the latter two were the independent variables of interest.

Separate general linear model regressions were run measuring for the dependent variables (surface area [55], cortical thickness [56], and volume). Variables were assessed for normality. Analyses were done separately between each hemisphere (right and left). For example, sex, VO_2_, and sex*VO_2_ parameters were run by fitting a regression at each vertex to predict left whole-brain surface area, and so on for each metric of morphometry for both hemispheres. Corrections for multiple comparisons were made using Monte Carlo simulations at a cluster wise probability of p < .05 and correcting across both hemispheric spaces. All decisions about statistical significance were made if p < .05. Regions that met statistical significance were annotated using the Desikan-Killiany Atlas. To confirm directionality of sex*VO_2_ interactions, any significant regions from the whole brain CT, SA, or volume analyses were extracted into SPSS. Correlations were then run between VO_2_ and ROI, separated by sex. Figures were produced using R package ‘fsbrain’ [57].

Follow-Up Intracranial Volume (ICV) Analyses. Estimated intracranial volume (ICV) was considered as a potential covariate in the primary analyses. Given recent evidence [58] in FreeSurfer that suggests correlation between ICV (which in FreeSurfer includes non-brain matter such as cerebrospinal fluid and fat) and total brain volume, suggesting a significant issue of multicollinearity, the decision was made *a priori* to not include ICV as an additional covariate in primary analyses. The primary concerns are regarding sex differences in ICV; however, simple sex differences were not the primary focus. Rather, we were most interested in the interaction between sex and VO_2_ maximum. Notably, neither high fit v. low fit groups (p = .29) nor males and females (p = .60) differed by ICV, nor was VO_2_ maximum performance correlated with ICV (p = .31). However, given this is a debated area and others (e.g., [59]) include ICV as a covariate in volume-based (i.e., volume, SA) investigations, analyses were re-run with the addition of ICV as a covariate to improve reproducibility and comparison across the field. In these analyses, sex, VO_2_ levels, sex-by-VO_2_, and ICV were included.

## Results

### Demographics

Fitness groups were used for descriptive purposes; they did not differ significantly by sex, race, ethnicity, age, or education (see Table 1). As expected, they did differ by body fat percentage (t(61) = 2.87, p = .006) and BMI (t(61) = 2.30, p = .026). There were also no significant differences between sex by race, ethnicity, age, or education (see Table 2).

**Table 1:** Demographics, substance use, and fitness characteristics by fitness group.

	% or *M* (SD) Range (n = 63)
Age	21.16 (2.5) 16–25
Education	14.41 (2.23) 9–21
Sex (% female)	51%
% Caucasian	69%
Asian	n = 6
Native Hawaiian/Other Pacific Islander	n = 1
Black or African American	n = 5
White or Caucasian	n = 44
More than one race	n = 6
Unknown	n = 1
% Hispanic/Latino/a	10%
VO_2_ Peak (ml/kg/min)	42.04 (9.44) 24.5–62.9
Body Fat %	21.52 (9.91) 3.4–47.2
Height (inches)	67.06 (3.87) 59–76.5
Weight (lbs)	153.28 (29.71) 103.4–263.6
BMI	24.04 (4.60) 17.4–39.1
Past Year Alcohol Use (Standard Drinks)	163.33 (226.42) 0–883
Past Year Cigarette Use (Cigarettes)	55.35 (222.89) 0–1165
Past Year Cannabis Use (Joints)	11.46 (24.28) 0–92.10

Notes: M = mean; SD = standard deviation.

**Table 2:** Demographics, substance use, and fitness characteristics by sex.

	Female (n = 32) % or *M* (SD) Range	Male (n = 31) % or *M* (SD) Range
Age	21.5 (2.53) 16–25	20.81 (2.60) 16–25
Education	14.53 (2.11) 11–21	14.29 (2.38) 9–19
% Caucasian	63%	77%
Asian	n = 1	n = 5
Native Hawaiian/Other Pacific Islander	n = 1	n = 0
Black or African American	n = 5	n = 0
White or Caucasian	n = 20	n = 24
More than one race	n = 4	n = 2
Unknown	n = 1	n = 0
% Hispanic/Latino/a	16%	3%
*VO_2_ Peak (ml/kg/min)	37.14 (7.99) 24.5–60.1	47.10 (8.12) 28.6–62.9
*Body Fat %	28.38 (7.28) 16.3–47.2	14.43 (6.78) 3.4–33.7
*Height (inches)	64.06 (2.07) 59–68	70.22 (2.47) 65.50–76.50
*Weight (lbs)	143.39 (26.49) 103.4–227.8	161.05 (30.31) 117.4–263.6
BMI	24.68 (4.77) 18–39.1	22.93 (4.19) 17.4–35.8
Past Year Alcohol Use (Standard Drinks)	125.81 (208.49) 0–883	201.65 (241.13) 0–756.5
Past Year Cigarette Use (Cigarettes)	48.05 (208.75) 0–1165	62.89 (239.84) 0–992.50
Past Year Cannabis Use (Joints)	10.23 (24.55) 0–92.10	11.76 (23.60) 0–81.17

Notes: M = mean; SD = standard deviation.

*p < .05.

#### Aerobic fitness

Participants on average had a VO_2_ level of 42.0ml/kg/min (SD = 9.4. Min = 24.5, Max = 62.9). Males had significantly higher VO_2_ levels than their female counterparts (t(61) = 4.9, p < .001). Further, participants on average had a body fat percentage of 21.5% (SD = 9.9, Min = 3.4, Max = 47.2). Female participants had significantly higher rates of body fat percentage compared to male participants (t(61) = 2.46, p = .017). Further, females had significantly lower height (t(61) = 10.75, p < .001) and weight (t(61) = 2.46, p = .017) compared to males. A Pearson correlation between VO_2_ peak level and body fat percentage shows a strong negative relationship between VO_2_ levels and body fat (r = -0.65), such that high VO_2_ is highly associated with lower body fat percentage. Due to the overlap of variance between these two variables creating multicollinearity, we did not incorporate body fat percentage in our analyses.

### Primary imaging results

Full results are presented in Table 3.

**Table 3:** Morphometrical findings.

	*t*	Size (mm^2^)	x	y	z	*p*
*Cortical Thickness*						
**VO**_**2**_ **Finding**						
Left Lateral Occipital	-3.771	2497.2	-20.7	-98.1	11.5	0.0002
Left Superior Parietal	-3.339	1129.52	-34.2	-48	58.8	0.00559
Left Cuneus	-2.929	921.61	-11.8	-71.6	16.8	0.02208
Right Precuneus	-3.189	1174.84	22.4	-61	23.8	0.0038
Right Lateral Occipital	-3.074	1616.07	18.7	-97.5	14.4	0.0002
Right Lateral Occipital (2)	-3.043	1299.54	18.8	-89.5	-6.4	0.0014
Right Inferior Parietal	-2.871	918.89	32.1	-62.2	46	0.0284
*Volume*						
**VO**_**2**_ **Finding**						
Left Lateral Occipital	-2.99	1326.89	-15.9	-94.2	-10.6	0.0028
**Gender Finding**						
Left Rostral Anterior Cingulate	3.972	1497.89	-7	35.5	0.0	0.0004
Left Lateral Occipital	3.09	1799.79	-35.4	-88.6	-13.2	0.0002
Right Superior Frontal	4.337	944.03	13	7.7	38.8	0.0482
*Surface Area*						
**VO**_**2**_ **Finding**						
Left Inferior Parietal	3.692	2390.2	-44.1	-63.5	10.8	0.0014
Right Inferior Parietal	4.743	2263.23	32.5	-64.4	39.4	0.0014
**Gender Finding**						
Left Inferior Parietal	3.48	3729.01	-38.6	-48.7	34.5	0.0002
Left Rostral Anterior Cingulate	3.123	3997.89	-5.9	25.5	-6.2	0.0002
Left Fusiform	3.02	2143.9	-32	-53.9	-9.6	0.0036
Right Caudal Anterior Cingulate	4.007	4482.93	11.8	10.8	36	0.0002
Right Superior Parietal	3.197	2611.88	31.5	-36	40.8	0.0002
Right Fusiform	2.92	2833.28	31.9	-57.3	-9.9	0.0002
**VO**_2_*Gender Finding						
Left Inferior Parietal	-2.834	1800.38	-38.3	-48.7	34.2	0.01475
Right Paracentral	-3.687	2248.47	13.9	-12.6	43.7	0.0014
Right Supramarginal	-3.333	1749.1	31.7	-35.5	40.7	0.00958

#### Cortical thickness (mm)

VO_2_ performance was significantly related to cortical thickness in bilateral occipital regions (p < .001), left superior parietal (p = .005), right inferior parietal regions (p = .02), left cuneus (p = .02), and right precuneus regions of the brain (p = .004). Higher VO_2_ performance was associated with lower cortical thickness in these regions (see Fig 1). There were no significant differences in cortical thickness by sex or VO_2_ by sex interaction.

**Fig 1:** Cortical thickness. Higher VO_2_ is associated with thinner left lateral occipital, left superior parietal, left cuneus, right precuneus, right lateral occipital, and right inferior parietal regions. Clusters are labeled using the Desikan-Killiany atlas with effect size masked onto each significant cluster.

#### Volume (mm^3^)

There was a significant relationship between VO_2_ performance and volume in the left lateral occipital region of the brain (p = .002), where higher VO_2_ performance was related to lower volume. Males had significantly higher volume compared to their female counterparts in the left rostral anterior cingulate (p < .001), left lateral occipital (p < .001), and right superior frontal brain regions (p = .05) when controlling for VO_2_ performance (see Fig 2). There was not a significant interaction on volume between VO_2_ performance and sex.

**Fig 2:** Volume. Clusters are labeled using the Desikan-Killiany atlas. (a) Posterior and inferior view of left lateral occipital VO_2_ finding with the effect size masked onto the cluster. Higher VO_2_ is associated with lower volume in this region. (b) Males had larger volumes than females in the left rostral anterior cingulate (green), left lateral occipital (yellow), and right superior frontal (purple) regions.

#### Surface area (mm^2^)

There was a significant relationship between VO_2_ performance and surface area in bilateral regions of the inferior parietal (p = .001) with higher VO_2_ performance being associated with larger surface area. Males had significantly higher surface area compared to their female counterparts in bilateral areas of the fusiform (p < .01), left inferior parietal (p < .001), left rostral anterior cingulate (p < .001), right caudal anterior cingulate (p < .001), and right superior parietal regions of the brain (p < .001) when controlling for VO_2_ performance. There was a significant VO_2_ by sex interaction in the left inferior parietal (p = .02), the right paracentral gyrus (p = .002), and the right supramarginal (p < .01) regions of the brain. The interaction showed that higher VO_2_ performance was associated with increased surface area in these regions for female participants compared to their male counterparts (Fig 3).

**Fig 3:** Surface area. Scatter plot of sex-by-VO_2_ interaction observed in the (a) right paracentral, (b) right supramarginal, and (c) left inferior parietal regions. Higher VO_2_ performance was associated with increased surface area for female participants (red = female) compared to male participants (blue = male). (d) Sex-by-VO_2_ findings observed in right paracentral (purple), right supramarginal (green), and left inferior parietal (yellow) surface area, regions are labeled using the Desikan-Killiany atlas.

To confirm this interpretation of directionality for sex-by-VO_2_ interactions, data for significant ROIs were extracted into SPSS for correlation analysis of VO_2_ by ROI, separated by sex. In females, higher VO_2_ was correlated with higher SA in the left inferior parietal (r = .568, p = .001), right paracentral (r = .509, p = .003), and right supramarginal (r = .508, p = .003) regions. In contrast, in males, higher VO_2_ was correlated with lower SA in left inferior parietal (r = -.482, p = .006), right paracentral (r = -.385, p = .03), and right supramarinal (r = -.414, p = .02) regions.

#### Follow-Up ICV analyses

*Volume*. There was a significant main effect of VO_2_ on left lateral occipital lobe (p = .0002), where higher VO_2_ was associated with smaller volume, when covarying for ICV. There was no interaction between VO_2_ and sex in volume in any regions. *Surface Area*. There were no significant main effects or interactions in SA when ICV was included as a covariate.

## Discussion

Aerobic fitness level may be an important contributor to brain health and neurodevelopment. As such, we assessed three measures of cortical development (gray matter volume, cortical thickness, and surface area) in adolescents and young adults with varying levels of aerobic fitness. In independent regression analyses, we found aerobic fitness related to volume, surface area, and cortical thickness. Higher aerobic fitness level, measured by VO_2_ testing, was significantly related to thinner occipital, parietal, cuneus, and precuneus regions, reduced occipital volume, and larger parietal surface area. Further, an interaction was present between fitness and sex, such that higher fit females demonstrated larger surface area in frontal (paracentral gyrus) and parietal regions, with lower fitness in males being associated with larger surface area. These findings were present when not controlling for ICV in volume or SA analyses.

Consistent with prior findings of aerobic fitness in healthy adolescents [27], some of the most pronounced findings are within sensorimotor regions. Specifically, we found links between higher aerobic fitness level and thinner parietal and occipital cortices, larger parietal surface area, and reduced occipital volume. Neurodevelopment in these regions occurs broadly across all of adolescence into early adulthood [60]. Change in aerobic fitness following an aerobic exercise intervention similarly related to increased cortical thickness in parietal and precuneus regions in older adults [61], perhaps indicating these areas are uniquely susceptible to aerobic fitness level, with changes in directionality depending on age. As has been suggested by others [27], these neuroanatomical differences may also be related to greater engagement in sports behaviors which depend on quick sensory processing, leading to advanced maturation.

Sex differences exist across development in surface area and volume, but less so in cortical thickness [10,60]. Consistent with this, we found no difference in cortical thickness by sex, but that lower fit males had larger surface area in frontal and parietal regions than higher fit males, while higher fit females had larger surface area in these same regions, when ICV was not included as a covariate. Vijayakumar and colleagues (2016) found an independent effect of sex, with males demonstrating larger surface area and volume across the cerebral cortex than females, including in many of the regions found here. Notably, they did not assess for the influence of aerobic fitness level and their sample covered a younger and broader age range (11–20 years-old). In addition, age appears to have a significant effect in volumetric differences, potentially contributing to the lack of fitness by sex interactions here, as indicated by prior research in prepubescent youth who did not show the same sex differences in volume [26]. Thus, differences in structure are likely a combination of age, sex, and fitness level differences. It is also important to note that we found males demonstrated significantly higher VO_2_ performance. As aerobic fitness level demonstrated a main effect relationship to morphometry, it may be that males’ unique neuroanatomical pattern may be due to their more robust aerobic fitness performance. As such, future research should assess differences by sex, while also accounting for potential developmental differences due to age and fitness, and carefully considering whether or not to include ICV as a control variable.

Despite hypothesizing a positive relationship between aerobic fitness level and brain volume, results suggest increased fitness level was linked with *reduced* left lateral occipital lobe volume when ICV was not included in analyses. Several possible reasons for this are noted. This may reflect superior pruning [62], leading to reduced volume. In addition, the differential direction of findings compared to other samples may be due to the inclusion of both males and females versus primarily male samples [25–28], as females tend to mature neurodevelopmentally slightly earlier than males [8,9]. Difference in methodology may also lead to apparently conflicting findings, as Herting and colleagues (2016) used a self-report measure of aerobic fitness while the present study utilized an objective, standardized method of aerobic fitness measurement. Finally, regions assessed differed (e.g., hippocampal and entorhinal cortex [29]; whole-brain here), which may contribute to the differing results. Still, combined with our prior study showing a link between higher aerobic fitness level and better cognitive performance [42], greater aerobic fitness appears to be advantageous for brain morphometry and function in physically healthy adolescents and young adults.

These suggested brain-behavior relationships are consistent with previous research that found regular exercise is also linked to better visual perceptual learning in adults (Connell, 2018), and improved executive functioning in emerging adults [63–65]. Engagement in aerobic activity has also resulted in acute changes in activation patterns in sensorimotor and occipital regions in young adults [66] and endurance athletes [67]. Thus, these underlying neuroanatomical changes may relate to functional improvements in high-fit adolescents and young adults. Consistent with this, other work by our group does show being more aerobically fit is related to better working memory and selective attention regardless of sex, and better sustained attention in more fit males (Wade et al., under review); however, these behavioral differences have not be examined in relation to underlying neuroanatomical structure. Given the limited sample size and power of the present analyses, we are currently unable to investigate these brain-behavior relationships in this sample. However, large-scale longitudinal studies in adolescents and young adults, such as the Adolescent Brain Cognitive Development (ABCD) study, will help clarify these relationships while also controlling for potentially confounding factors such as body fat distribution.

Multiple underlying neuromechanisms may lead to earlier maturation in aerobically fit emerging adults. Aerobic fitness is known to increase following aerobic exercise [61]. Growth factors (e.g., BDNF) [14,16,17,19,68] and neurogenesis [12,13] increase in response to exercise. Decreased neuroinflammation [14,22,69] and improved cathecholaminergic function [21,70,71] also both likely lead to healthier brain development. Of course, these studies investigated aerobic exercise rather than fitness level, as assessed here. Future studies should assess aerobic fitness level, rather than only exercise, to determine whether these mechanisms may be contributing to the present findings.

Volume-based analyses may be vulnerable to differences due to head size or intracranial volume. This has led to a debate regarding whether it is appropriate to include ICV estimates in volume and surface area analyses and the suggestion that its inclusion needs to be carefully considered [58,72]. Others have previously determined not to include ICV if there is no group difference by sex or fitness in ICV [27], as demonstrated in the present sample. Therefore, it was decided *a priori* not to include ICV in our primary analyses. At the same time, several large studies have recently included ICV and found it an important covariate ([59], see [73]). Interestingly, as the present primary results without ICV found specific regional differences rather than significant differences in clusters throughout the whole brain as might be expected if it was a total volume issue, it may be less likely that ICV has a significant impact on the present results. On balance and consistent with a recent review documenting both ICV and non-ICV controlled findings [73], volume and SA analyses are changed when ICV is included as a covariate, suggesting continued replication of structural neuroimaging findings and caution in interpretation is needed.

Results here are notable for the use of objective measurement of aerobic fitness, novel investigation of sex, and for multiple measures of brain morphometry. As with all research, however, limitations should be considered. As a cross-sectional study, causality cannot be established, and longitudinal studies of change in aerobic fitness level are needed to determine directionality. While sex is an important moderator of many outcomes, other factors (e.g., genetic variations, such as in BDNF) have previously been shown to relate to different morphology [27] and need combined consideration in the future. As the sample recruited had to be physically healthy, without psychiatric diagnoses, aerobic fitness may differently influence individuals with physical or mental health difficulties. Thus, results here are likely comparable in many healthy emerging adults recruited within the community, though we also note this sample is fairly well educated and predominately white, limiting generalizability.

Here the relationships between aerobic fitness and brain structure in male and female adolescents and young adults were examined. Results indicated that aerobic fitness level was associated with signs of earlier neuromaturation (decreased gray matter volume, decreased cortical thickness, and increased surface area) in sensorimotor and occipital regions without ICV as a covariate. In addition, sex interacted with fitness level, as higher-fit males demonstrated lower surface area in frontal and parietal regions, while higher fit females showed higher surface area. Taken together, results suggest aerobic fitness level may be an important contributor to neurodevelopment through emerging adulthood. Further, the impact of aerobic fitness on brain structure may be moderated by sex. Future studies will need to examine these relationships longitudinally and determine whether the impact of aerobic fitness interventions on neurocognitive outcomes are moderated by sex.

## Supporting information

S1 File (SAV)
